The article "Hirudin promotes proliferation and osteogenic differentiation of HBMSCs via activation of cyclic guanosine monophosphate (cGMP)/protein kinase-G (PKG) signaling pathway" was published in 2022. Journal: Bioengineered.

# Hirudin promotes proliferation and osteogenic differentiation of HBMSCs via activation of cyclic guanosine monophosphate (cGMP)/protein kinase-G (PKG) signaling pathway

**DOI:** 10.1080/21655979.2021.2008697

**Published:** 2022-02-24

**Authors:** Shun Cao, Xianghui Li, Ting Feng, Yaqing Li, Hongwei Ding, Lin Xie, Quanhong Yang

**Affiliations:** a Department of Orthopaedics, The Second Affiliated Hospital of Nanjing University of Chinese Medicine, Nanjing City, PR China; b Department of General Studies, Affiliated Hospital of Shaanxi University of Traditional Chinese Medicine, Xianyang City, PR China; c Academic Affairs Office, Jiangsu Health Vocational College, Nanjing City, PR China; d Department of Orthopedics, Jiangsu Province Integrated Traditional Chinese and Western Medicine Hospital, Nanjing City, PR China

**Keywords:** Osteoporosis, Hirudin, cell proliferation, osteogenic differentiation, human bone marrow-derived mesenchymal stem cells, cGMP

## Abstract

Osteoporosis is a public health problem resulting in higher susceptibility to bone fracture. Hirudin is known as a direct thrombin inhibitor, which is isolated from the salivary gland of the medicinal leech. The present study aimed to evaluate the effect of Hirudin on the proliferation and osteogenic differentiation of human bone marrow-derived mesenchymal stem cells (HBMSCs). In our study, the effect of Hirudin on the proliferation of HBMSCs was evaluated with the CCK-8 and MTT assays. The capacity of osteogenic differentiation and mineralization of HBMSCs was evaluated with ALP and alizarin red staining, respectively. cGMP content was determined by ELISA. Western blotting and qRT-PCR were used to investigate the effect of Hirudin on the expression of osteoblast-specific markers, including Runx2, osterix (OSX), osteocalcin (OCN), and collagen1 (Col1). In our study, Hirudin treatment promoted cell viability. Moreover, Hirudin treatment increased ALP activity of HBMSCs and red coloration of alizarin. Interestingly, cGMP inhibitor partly reversed the effect of Hirudin on the proliferation, differentiation and mineralization of HBMSCs. In conclusion, Hirudin promoted the proliferation, differentiation and mineralization of HBMSCs via activation of cGMP signaling pathway. Hence, Hirudin contributed to bone remodeling and might represent as an effective agent for the treatment of osteoporosis.

## Introduction

Osteoporosis is one of the public health problems in the elderly population and postmenopausal females, characterized by low bone mass and deteriorated bone structure in bone tissue [1]. The imbalance between bone formation and resorption contributes to the onset and development of osteoporosis, resulting in higher susceptibility to bone fracture [2,3]. Adult stem cells used for bone tissue engineering include bone marrow stem cells (BMSCs), adipose-derived stem cells (ASCs), and dental pulp stem cells. BMSCs are most frequently used in bone tissue engineering because of their high osteogenic differentiation potentials [4]. Human bone marrow-derived mesenchymal stem cells (HBMSCs), known as multipotent cells, have the potential to differentiate into various connective tissue cell types including osteogenic, chondrogenic and adipogenic lineages [5]. It is well established that mesenchymal stem cells (MSCs) can move to the fracture sites and differentiate into osteocytes for bone healing [6]. Hence, enhancing the osteogenic differentiation ability of HBMSCs may be a promising therapeutic strategy for osteoporosis treatment.

The article "Hirudin promotes proliferation and osteogenic differentiation of HBMSCs via activation of cyclic guanosine monophosphate (cGMP)/protein kinase-G (PKG) signaling pathway" was published in 2022. Journal: Bioengineered.

Hirudin, a direct thrombin inhibitor, is isolated from the salivary gland of the medicinal leech *Hirudo medicinalis*, which is involved in multiple pharmacological activities including anti-cancer, anti-coagulation and anti-hyperlipidemia effects. Numerous studies have shown that Hirudin plays a vital role in many diseases, such as human glioma [7], diabetic cataract [8] and Alzheimer’s disease [9]. However, the effect of Hirudin on the proliferation and osteogenic differentiation of HBMSCs has not been clarified. Interestingly, Kazuhiko et al. have suggested that thrombin has a stimulated effect on the synthesis of interleukin‑6 (IL‑6) [10]. It has reported that IL-6 negatively regulates osteoblast differentiation through MEK2 and Akt2 signaling [11]. Moreover, Melagatran, a novel group of thrombin inhibitors, may help prevent heparin-induced inhibitory effects on human osteoblasts [12]. Hence, we hypothesize that Hirudin may have potential application in preventing bone deficiency.

In the literature, icariin is found to exert stimulatory effects on osteogenic differentiation, which is mediated by PI3K-AKT-endothelial NO synthase (eNOS)-nitric oxide (NO)-cyclic guanosine monophosphate (cGMP)-protein kinase-G (PKG) signaling pathway [13]. Moreover, previous studies have reported that the proliferation and osteoblastic differentiation of HBMSCs, regulated by NO/cGMP pathway, is helpful for bone formation and thus prevents osteoporosis [14]. Importantly, Kobsar et al. have demonstrated that two thrombin inhibitors (Hirudin and lepirudin) induce the activation of the soluble guanylyl cyclase (sGC) and the cGMP signaling pathways in washed human platelets [15]. Thus, we assumed that cGMP/PKG signaling pathways may be involved in the effect of Hirudin on osteoblasts.

Therefore, in this paper, we examined the effects of Hirudin on the proliferation and osteogenic differentiation of HBMSCs and discussed the specific mechanisms involved. It provided a theoretical basis for Hirudin in the clinical treatment of osteoporosis.

The article "Hirudin promotes proliferation and osteogenic differentiation of HBMSCs via activation of cyclic guanosine monophosphate (cGMP)/protein kinase-G (PKG) signaling pathway" was published in 2022. Journal: Bioengineered.

## Materials and methods

### Cell culture

Human bone marrow-derived mesenchymal stem cells (HBMSCs, SALILA, Guangzhou, China) were maintained in Dulbecco’s modified Eagle’s medium (Gibco, Carlsbad, CA, USA) with 10% fetal bovine serum (FBS) in a humidified incubator at 37°C with 5% CO_2_. The HBMSCs were maintained with osteogenic differentiation induction medium (OM) with 100 mM dexamethasone, 0.05 mM ascorbic acid, and 10 mM β-glycerophosphate for osteogenic induction. The medium was changed every 48 h. The cells were divided into control group, OM group and OM+Hirudin group (10, 20, 40, 80 and 160 μg/mL). The concentrations of Hirudin were 10, 20, 40, 80 and 160 μg/mL, and the cells were treated for 48 h. Hirudin at a concentration of 80 μg/mL was selected for subsequent experiments. Then, the mechanism of Hirudin affecting cell proliferation and osteogenic differentiation was discussed, 50 μM Rp-8-Br-cGMP (cGMP/PKG inhibitor) was used to pre-treat cells for 30 min and the cells were divided into OM group, OM+80 μg/mL Hirudin group and Rp-8-Br-cGMP+OM+80 μg/mL Hirudin group.

### Cell counting kit-8 (CCK-8) assay

HBMSCs in the logarithmic growth phase were incubated in 96-well plates at a density of 5 × 10^3^/well for 24 h at 37°C. The cells were divided into control group, OM group and OM + Hirudin group (10, 20, 40, 80 and 160 μg/mL). Proliferation data are presented as means ± SD. Cell viability was estimated at 48-h treatment with 100 μL osteogenic medium containing 10, 20, 40, 80 or 160 μg/mL Hirudin, and then, 10 μl CCK-8 solution (Dojindo, Kumamoto, Japan) was added to each well, followed by incubation for 1 h. The absorbance value was recorded at 450 nm.

### MTT assay

HBMSCs in the logarithmic growth phase were incubated in 96-well plates at a density of 5 × 10^3^/well and cultured with a basal medium or osteogenic medium containing Hirudin (80 μg/mL) or pre-treated with 50 μM Rp-8-Br-cGMP (cGMP inhibitor) for 30 min for 1, 3, 7 and 14 days, respectively. The cells were then incubated with 20 μl MTT (5 mg/mL, Amresco, USA) solution at 37°C for 4 h at 1D, 3D, 7D and 14D. Subsequently, the medium was replaced with the MTT formazan crystals and dissolved with 200 μl DMSO, and the absorbance value was at last recorded at 450 nm using a microplate reader (Spectra Max M2e Microplate Reader; Molecular Devices Corporation, Sunnyvale, CA, USA).

### Alkaline phosphatase (ALP) staining

HBMSCs in the logarithmic growth phase were cultured in 6-well plates (2.0 × 10^5^ cells/well). After the Hirudin treatment for 48 h, ALP staining was performed on HBMSC lysates, which was carried out in accordance with the instructions of the commercial ALP assay kit (MKBio, Shanghai, China). Cell observation was done under a light microscope (Carl Zeiss, Jena, Germany, magnification ×200) at last. The absorbance of the cell culture was measured at 405 nm, and the final calcium level was normalized according to the total protein concentration in duplicate plates [16].

The article "Hirudin promotes proliferation and osteogenic differentiation of HBMSCs via activation of cyclic guanosine monophosphate (cGMP)/protein kinase-G (PKG) signaling pathway" was published in 2022. Journal: Bioengineered.

### Alizarin red staining

HBMSCs in the logarithmic growth phase were cultured in 6-well plates (2.0 × 10^5^ cells/well). After induction, HBMSCs were cultured in 24-well plates and fixed with 97% ethanol, rinsed with ddH_2_O, and then stained with 2% alizarin red staining solution (adjusted to pH 4.2) for 10 min. Subsequently, the stained HBMSCs were captured under an inverted fluorescence microscope (Olympus, Japan, magnification ×200) [17].

### Quantitative real-time polymerase chain reaction (qRT-PCR)

Total RNA was extracted by means of TRIzol® reagent (Thermo Fisher Scientific, Inc.) according to the suppliers’ instructions and was reverse-transcribed into cDNA using Hifair® III 1st Strand cDNA Synthesis SuperMix for qPCR (Yeasen, Shanghai, China). cDNA (1 μL) was taken as the template for real-time PCR, and the reaction conditions were as follows: 95°C for 10 min, 95°C for 15 s, 60°C for 30 s, 72°C for 30 s, and total 35 cycles. The relative quantity of gene expression was calculated with 2^–∆∆Ct^ method [18] and normalized to GAPDH expression. The primer sequences are presented as follows: Runx2: forward 5ʹ-CTAGGCGCATTTCAGGTGCT-3ʹ, reverse 5ʹ-TGGCAGGTAGGTGTGGTAGT-3ʹ;osterix (OSX): forward 5′-GCCTACTTACCGTGACTTT-3′, reverse 5′-GCCCACTATTGCCAACTGC-3′; osteocalcin (OCN): forward 5ʹ-GCCCGAGACTTTGAGAAGAACTAC-3ʹ, reverse 5ʹ-GATGTCCTGCTCCTTGATGC-3ʹ; collagen1 (Col1): forward 5ʹ-GACATGTTCAGCTTTGTGGACCTC-3ʹ, reverse 5ʹ-GGGACCCTTAGGCCATTGTGTA-3ʹ; and GAPDH:forward5ʹ-GGAGCGAGATCCCTCCAAAAT-3ʹ,reverse5ʹ-GGCTGTTGTCATACTTCTCATGG-3ʹ.

### Western blotting

After the cells in different groups were digested, centrifuged and lysed, the total proteins were isolated for detection of protein concentration. 30 μL protein samples were fractionated by corresponding 12% SDS-PAGE gel and then transferred onto PVDF membranes. After incubation with antibodies against PKG (1:1000), Runx2 (1:1000), OSX (1:1000), OCN (1:1000), Col1 (1:1000), and GAPDH (1:2000) overnight at 4°C, the membranes were incubated with appropriate HRP-conjugated secondary antibody for 2 h before ECL color development. The relative quantity of protein expression in different groups was calculated using ImageJ software.

The article "Hirudin promotes proliferation and osteogenic differentiation of HBMSCs via activation of cyclic guanosine monophosphate (cGMP)/protein kinase-G (PKG) signaling pathway" was published in 2022. Journal: Bioengineered.

### ELISA

HBMSCs in the logarithmic growth phase were incubated in 96-well plates at a density of 5 × 10^3^/well for 24 h at 37°C. The concentrations of cyclic guanosine monophosphate (cGMP) and PKG in supernatants of HBMSCs with Hirudin treatment for about 48 h were quantified by using the Cyclic GMP Complete ELISA Kit (Abcam Cambridge, United Kingdom), according to the manufacturer’s protocols. The absorbance (A450) was detected by a microplate reader.

### Statistical analysis

All assays were carried out in triplicate, and all values are presented as the mean ± standard deviation (SD). Differences between the two groups were analyzed using Student’s *t* test, and differences among multiple groups were analyzed using one-way ANOVA followed by Tukey post hoc test. A value of *P* <0.05 was considered statistically significant.

## Results

### Hirudin treatment promoted cell proliferation

Firstly, the cellular cytotoxicity of Hirudin was measured after multiple doses of Hirudin treatment for 48 h. The results from CCK-8 assay demonstrated that 160 μg/mL Hirudin significantly suppressed the viability of HBMSCs. Hence, 80 μg/mL Hirudin was selected for further study (Figure 1a).

**Figure 1.** Hirudin treatment promoted cell viability. (a) The cytotoxicity of HBMSCs treated for 48 h by Hirudin was evaluated with the CCK-8 assay. (b) The proliferation of HBMSCs treated for 48 h by Hirudin was evaluated with the MTT assays. Error bars represent the mean ± SD from three independent experiments. ***P < 0.001 *vs*. Control. ^#^*P* < 0.05, ^###^*P* < 0.001 *vs*. OM.

To explore the effect of Hirudin on the development of osteoporosis, the proliferation of HBMSCs was determined by MTT assay. At the indicated time (1, 3, 7 and 14 days), we found that Hirudin treatment promoted cell proliferation in a time-dependent manner (Figure 1b). These results suggested that Hirudin treatment promoted the proliferation of HBMSCs.

### Hirudin treatment promoted the differentiation and mineralization of HBMSCs

To further investigate the effect of Hirudin on the development of osteoporosis, the differentiation and mineralization of HBMSCs were detected by ALP staining and alizarin red staining, respectively. As shown in Figure 2a, Hirudin treatment significantly increased the ALP activity of HBMSCs. Alizarin red staining manifested that the red coloration of alizarin was notably increased in OM + 80 μg/mL Hirudin group compared with control or OM group (Figure 2b). Moreover, the protein and mRNA levels of Runx2, OSX, OCN, and Col1 were upregulated by Hirudin treatment compared with control or OM group (Figure 2c-e). These results indicated that Hirudin treatment promoted the differentiation and mineralization of HBMSCs.

The article "Hirudin promotes proliferation and osteogenic differentiation of HBMSCs via activation of cyclic guanosine monophosphate (cGMP)/protein kinase-G (PKG) signaling pathway" was published in 2022. Journal: Bioengineered.

**Figure 2.** Hirudin treatment increased ALP activity of HBMSCs and red coloration of alizarin. (a) The capacity of osteogenic differentiation of HBMSCs treated for 48 h by Hirudin was evaluated by ALP staining and a bar graph is a statistical analysis of the image. (b) The capacity of mineralization of HBMSCs treated for 48 h by Hirudin was determined by alizarin red staining and a bar graph is a statistical analysis of the image. (c) The protein levels of osteoblast-specific markers, including Runx2, osterix (OSX), osteocalcin (OCN), and collagen1 (Col1), were quantified by Western blotting and quantification (d). (e) The relative mRNA levels of Runx2, OSX, OCN and Col1 were quantified by qRT-PCR. Error bars represent the mean ± SD from three independent experiments. **P < 0.01, ***P < 0.001 *vs*. Control. ^##^*P* < 0.01, ^###^*P* < 0.001 *vs*. OM.

### The inhibitor of cGMP/PKG partly reversed the effect of Hirudin on the proliferation, differentiation and mineralization of HBMSCs

To investigate the underlying mechanism of Hirudin in osteoporosis development, the cGMP/PKG inhibitor was applied. After cells were treated with 50 μM Rp-8-Br-cGMP (cGMP inhibitor) for 30 min combined with Hirudin treatment, the proliferation, differentiation and mineralization of HBMSCs were examined again, as described above. The result from ELISA showed that the cGMP concentration was remarkably enhanced by Hirudin treatment compared with control or OM group (Figure 3a). Western blot results showed that compared with OM group, the expression of PKG was increased obviously in OM+80 μg/mL Hirudin group (Figure 3b). MTT assay demonstrated that cGMP/PKG inhibitor abolished the promoting effect of Hirudin treatment on HBMSC proliferation (Figure 4a). Furthermore, cGMP/PKG inhibitor also partly reversed the promoting effect of Hirudin treatment on the red coloration of alizarin and ALP activity of HBMSCs in OM + 80 μg/mL Hirudin group (Figure 4b-c). Moreover, the treatment of cGMP/PKG inhibitor led to a reduction in the expression of Runx2, OSX, OCN, and Col1 even under the condition of Hirudin treatment (Figure 4d-f). These results suggested that Hirudin treatment promoted the proliferation, differentiation and mineralization of HBMSCs via activation of cGMP/PKG signaling pathway.

**Figure 3.** Hirudin treatment elevated cGMP concentration in HBMSCs. (a) cGMP in supernatants of HBMSCs with Hirudin treatment for about 48 h was determined by ELISA. (b) Western blot detected the expression of PKG. Error bars represent the mean ± SD from three independent experiments. **P < 0.01 *vs*. Control. ^###^*P* < 0.001 *vs*. OM.

The article "Hirudin promotes proliferation and osteogenic differentiation of HBMSCs via activation of cyclic guanosine monophosphate (cGMP)/protein kinase-G (PKG) signaling pathway" was published in 2022. Journal: Bioengineered.

**Figure 4.** The inhibitor of cGMP partly reversed the effect of Hirudin on proliferation, differentiation and mineralization of HBMSCs. (a) The proliferation of OM induced HBMSCs pre-treated with Rp-8-Br-cGMP for 30 min and with Hirudin for 48 h was evaluated with the MTT assays. (b) The capacity of osteogenic differentiation of OM induced HBMSCs pre-treated with Rp-8-Br-cGMP for 30 min and with Hirudin for 48 h was evaluated by ALP staining. (c) The capacity of mineralization of OM induced HBMSCs pre-treated with Rp-8-Br-cGMP for 30 min and with Hirudin for 48 h was determined by alizarin red staining. (d) The protein levels of osteoblast-specific markers, including Runx2, osterix (OSX), osteocalcin (OCN), and collagen1 (Col1), were quantified by Western blotting and quantification (e). (f) The relative mRNA levels of Runx2, OSX, OCN and Col1 were quantified by qRT-PCR. Error bars represent the mean ± SD from three independent experiments. *P < 0.05, ***P < 0.001 *vs*. OM. ^#^*P* < 0.05, ^##^*P* < 0.01 *vs*. OM+80 μg/mL Hirudin.

## Discussion

Osteoporosis is defined as a systematic skeletal disease featured by decreased bone mineral density and damaged bone structure due to the imbalance between bone formation and resorption [19]. Rapidly accumulating evidence now suggests that HBMSC decline and osteoblastic differentiation deficiency can be defined as the important factors leading to osteoporosis [20,21]. Therefore, the improvement of proliferative and differentiative capacities of HBMSCs is believed to be a novel and effective strategy for osteoporosis treatment.

Natural Hirudin plays a crucial role in blood rheology improvement by inhibiting blood coagulation and thus has been extensively applied in China [22,23]. Most importantly, Hirudin is developed and represented as a promising agent and may probably replace heparin in clinical treatment in the future, due to the side effect of unfractionated heparin in osteoporosis treatment [24]. In our study, it was found that the treatment of Hirudin promoted cell proliferation in a time-dependent manner, suggesting that Hirudin played a regulative role in the proliferative capacity of HBMSCs. Interestingly, it was also found that Hirudin treatment promoted the differentiation and mineralization of HBMSCs and upregulated the protein levels of Runx2, OSX, OCN, and Col1. The proteins, including Runx2, OSX, OCN and Col1, were the most widely used osteoblast-specific markers for the detection of HBMSC differentiation [25,26]. Take RUNX2 as an example, as a key regulator of osteoblast differentiation, RUNX2 plays a crucial role in development and ossification of normal skeletons [27]. These findings revealed that Hirudin treatment promoted the proliferation, differentiation and mineralization of HBMSCs.

The article "Hirudin promotes proliferation and osteogenic differentiation of HBMSCs via activation of cyclic guanosine monophosphate (cGMP)/protein kinase-G (PKG) signaling pathway" was published in 2022. Journal: Bioengineered.

Interestingly, our results in this study also demonstrated that Hirudin treatment significantly elevated the concentration of cGMP and PKG. Anna et al. have reported that Hirudin induces the activation of the cGMP/PKG pathway in washed human platelets, which is consistent with our results [15]. Meanwhile, we further investigated the molecular mechanism involved in the effect of Hirudin on the cellular behaviors of HBMSCs. Rp-8-Br-cGMP, cGMP inhibitor, was applied to downregulate the cGMP/PKG level. Rp-8-Br-cGMP works by binding to PKG as a competitive inhibitor but does not activate PKG, thus blocking the activation of the cGMP/PKG signaling pathway [28]. Our findings showed that cGMP inhibitor partly reversed the effect of Hirudin on the proliferation, differentiation and mineralization of HBMSCs, as well as the expression of osteoblast-specific markers. Previous study showed that increasing cGMP can increase bone anabolic signals and protect bone [29]. Stimulating intracellular cGMP level can promote osteoblast differentiation, and inhibiting PKG can inhibit osteoblast differentiation [30]. Hence, cGMP/PKG signaling is essential for bone remodeling. Furthermore, Ghania et al. have reported that cGMP-dependent protein kinase-2 plays a regulative role in bone mass and prevents diabetic bone loss through promoting osteoblast proliferation and bone formation rates [31]. Taken together, Hirudin promoted the proliferation, differentiation and mineralization of HBMSCs via activation of cGMP/PKG signaling pathway. Besides, since the molecular mechanisms involved in our study are complex, the specific target of Hirudin remains to be further explored.

There are also limitations in our article. We only conducted experiments in cells but did not verify our results in animals, and we will further verify our results in animals in future experiments. In addition, the induction time of Hirudin was only selected for 48 h in our experiment, so we should screen the induction time of Hirudin, which is also one of the limitations of our paper. We will further screen the induction time of Hirudin in future experiments.

## Conclusion

In summary, our findings suggested that Hirudin promoted the proliferation, differentiation and mineralization of HBMSCs via activation of cGMP signaling pathway, suggesting that Hirudin contributed to bone remodeling and might be represented as an effective agent for the treatment of osteoporosis.

## Research highlights

Hirudin promotes proliferation of HBMSCs

Hirudin promotes osteogenic differentiation of HBMSCs

Hirudin regulates the activation of cGMP signaling pathway
